The article "Application and extension of the UTAUT2 model for determining behavioral intention factors in use of the artificial intelligence virtual assistants" was published in 2022. Journal: Front Psychol.

# Application and extension of the UTAUT2 model for determining behavioral intention factors in use of the artificial intelligence virtual assistants

**DOI:** 10.3389/fpsyg.2022.993935

**Published:** 2022-10-18

**Authors:** María García de Blanes Sebastián, José Ramón Sarmiento Guede, Arta Antonovica

**Affiliations:** Business Economics, Rey Juan Carlos University, Madrid, Spain

**Keywords:** virtual assistants, UTAUT2, users' behavioral intentions, technology implementation, artificial intelligence

## Abstract

Virtual Assistants, also known as conversational artificial intelligence, are transforming the reality around us. These virtual assistants have challenged our daily lives by assisting us in the different dimensions of our lives, such as health, entertainment, home, and education, among others. The main purpose of this study is to develop and empirically test a model to predict factors that affect users' behavioral intentions when they use intelligent virtual assistants. As a theoretical basis for investigating behavioral intention of using virtual assistants from the consumers' perspective, researchers employed the extended Unified Theory of Acceptance and Use of Technology (UTAUT2). For this research paper, seven variables were analyzed: performance expectancy, effort expectancy, facilitating conditions, social influence, hedonic motivation, habit, and price/value. In order to improve consumer behavior prediction, three additional factors were included in the study: perceived privacy risk, trust, and personal innovativeness. Researchers carried out an online survey with 304 responses. The obtained sample was analyzed with Structural Equation Modeling (SEM) through IBM SPSS V. 27.0 and AMOS V 27.0. The main study results reveal that factors, such as *habit, trust*, and *personal innovation*, have a significant impact on the adoption of virtual assistants. However, on the other side, *performance expectancy, effort expectancy, facilitating conditions, social influence, hedonic motivation, price/value*, and *perceived privacy risk* were not significant factors in the users' intention to adopt this service. This research paper examines the effect of personal innovation, security, and trust variables in relation to the use of virtual assistants. It contributes to a more holistic understanding of the adoption of these intelligent devices and tries to fill the knowledge gap on this topic, as it is an emerging technology. This investigation also provides relevant information on how to successfully implement these technologies.

## Introduction

The most recent developments around digital technologies open new possibilities in the Human-to-machine interaction (Dix, 2017). Virtual assistants (VAs) are remarkable for their functionalities by providing close to real conversations with humans using interfaces, and by representing a human-like image that simulates social skills recreating personable qualities that interact with humans *via* imitation. Some human abilities that are commonly recreated or represented as communicative traits include speech recognition, feedback loop, and interacting with the tool of the exchange in a conversation (Cassell, 2000). Some known VAs in everyday activities, Alexa, Siri, Cortana, and Bixby, complete essential tasks: starting phone calls, reporting weather, processing math and calculations, playing music lists, and many more (Chattaraman et al., 2019; Robinson et al., 2019). Artificial Intelligence (AI) is providing the tools for VAs to offer advanced voice interfaces, and to allow users to carry an interaction *via* internet connection by using real speech. These VA platforms are integrated in consumer devices *via* smartphones and tablets, as well as *via* platforms for home entertainment, incorporating speakers, bots, and messenger platforms (Guzman, 2019). Workplace environment interfaces can include: functions *via* chatbots, graphic design, speech recognition, media publishing, video editing, and accounting, etc., and can be found in VAs. The most recent dissemination from devices powered by AI and integrated business software into market technology will provide a bottom line 4.2 billion devices, which is estimated to double in number to 8.4 billion in 2024 (Statista, 2022).

The article "Application and extension of the UTAUT2 model for determining behavioral intention factors in use of the artificial intelligence virtual assistants" was published in 2022. Journal: Front Psychol.

In this context, scholars in the Information Technologies area have created a framework of the UTAUT2 theory (Venkatesh et al., 2012), where any empirical information and collected data can be studied to apply in different fields with varying angles within the technology realm (Venkatesh et al., 2016). This approach, and growing interest in VAs, provides field research to understand factors that lead to VAs adoption. This growing interest on studying factors from a consumer decision-making side creates a number of rationales that allow for insightful predictions within the adoption segment (Yang and Lee, 2019; Hasan et al., 2021; Pitardi and Marriott, 2021). It seems that there are not enough studies framing the factors that are influencing, or directly or indirectly changing, everyday needs and expectations in order to evolve according to users' needs. This became apparent mainly after many changes drastically affected our standard of living and interactions, as those that occurred in Spain during and after the last global pandemic caused by COVID-19.

The model UTAUT2 is the base framework, with an emphasis on *Perceived Privacy Risk* and *Perceived Trust* as constructs taken into consideration. As a result, the theoretical model is improved by adding *Personal Innovation* to the seminal notions developed by Dinev and Hart (2006) for an integrated framework. The following research questions and objectives lead the study.

The article "Application and extension of the UTAUT2 model for determining behavioral intention factors in use of the artificial intelligence virtual assistants" was published in 2022. Journal: Front Psychol.

Research questions:

- What are the factors impacting behavioral intention in the process of use for VAs?
- What degree of trust, perceived privacy risk, and personal innovation can be measured from VA usage?

Objectives:

- To explore the factors included in the model UTAUT2 directly impacting user behavior around VAs.
- To add rationales from the model UTAUT2 impacting user behavior around VAs.
- To evaluate the model of behavioral user intention aligned with empirical data in correlation with guiding variables.
- To establish a preliminary guideline from intention to usage for plausible advances around this area.

The study is presented in 6 sections. Section 1 is the Introduction. Section 2 sets a Theoretical framework, before introducing the hypothesis linked to relevant variables from the theories applied in Section 3, Selected variables for the study. Next, Section 4, Methodology, sets research standards, including methods, data collection, and data analysis. In Section 5 presents results and discussion. In Section 6, Conclusions and implocations are explained, prior to Section 7, Limitations and future research which provides the scope and closing remarks.

## Theoretical framework

### Virtual assistants

The use of artificial intelligence is being developed in line with the improvement of technology and tasks relating to AI implementations (Saad et al., 2017; Yang and Lee, 2019; Lopatovska et al., 2021). AI implementation in VA consumer devices, also called voice assisted tools, revolves around integrated data in IoT applications. These communicate with users, *via* speech, text, facial recognition, and gestures (Laranjo et al., 2018) to allow user interaction *via* natural language (Stieglitz et al., 2018). These devices are designed to provide a similar-to-human environment, having improved voice activated technology from the previous generation of devices; and due to the additional learning capability from input for a better performance, this technology has advanced a step further in its potential for personalization (Bawack et al., 2021; Vimalkumar et al., 2021). In general, the latest generation of voice assisted devices offers better-quality tools for services providing added space for personalization with regard to previous interactions (McLean and Osei-Frimpong, 2019; Pantano and Pizzi, 2020). Accordingly, digital adaptations in voice assisted devices extend on the expectation for performance and productivity in the workplace, so their link to hedonic pleasure and utility derived from usage has an impact on the balance that its users attain in their personal lives (Mishra et al., 2021; Jain et al., 2022). Popular personal assistant devices in the present-day marketplace, such as, Siri, Alexa, Cortana, and Bixby, are integrating common every day-use devices in consumer technology, such as speakers, autonomous vehicles and mobile devices, by integrating voice recognition into AI, so users interact with smartphones from a creative, novel, and more immediate interface. In recent years, VAs with integrated AI functionalities have been a leading trend in consumer technology due to the potential benefits derived from personalization, both in the workplace and in the home, and for the ease of use and added capabilities, which, in turn, create a positive feeling around VAs (Moriuchi, 2019).

The article "Application and extension of the UTAUT2 model for determining behavioral intention factors in use of the artificial intelligence virtual assistants" was published in 2022. Journal: Front Psychol.

### UTAUT2

The analysis of factors in technology adoption are core to research studies in the field for a great number of authors. The UTAUT model was derived *via* an evolved model from at least eight developments from different fields of study, pinning down technological change and adoption: Innovation Diffusion Theory IDT (Rogers, 1961); Theory of Reasoned Action TRA (Ajzen and Fishbein, 1980); Theory of Planned Behavior TPB (Ajzen, 1991); Social Cognitive Theory SCT (Bandura, 1986); Technology Acceptance Model TAM (Davis, 1989); Model of PC Utilization MPCU (Thompson et al., 1991); Motivational Model MM (Davis et al., 1992); C-TAM; Combined TAM-TPB (Taylor and Todd, 1995). The main value of this model arises from bringing a historic light in technology use by working around a set of constructs; that is, concepts that encapsulate what is central to the effects of technology use from a user's intention perspective (Yu, 2012). The UTAUT model centered on four constructs: *Performance Expectancy, Effort Expectancy, Social Influence*, and *Facilitating Conditions* with moderating demographic inputs: gender, age, level of expertise (experience), and perceived usefulness (Venkatesh et al., 2003). From these eight variables, a wrapping theory with their activated items from constructs, are presented in Table 1.

**Table 1:** Core constructs of UTAUT.

**Constructs**	**Variables**	**Model contributing to constructs**
Performance expectancy	Perceived usefulness	Technology Acceptance Model (TAM) 1–3; Combined TAM-TPB (Theory of Planned Behavior)
	Extrinsic motivation	Motivation Model (MM)
	Job-fit	Model of PC Utilization (MPCU)
	Relative advantage	Innovation Diffusion Theory (IDT)
	Outcome expectations	Social Cognition Theory (SCT)
Effort expectancy	Perceived ease of use	TAM 1–3
	Complexity	MPCU
Social influence	Subjective norms	TRA, TAM2, TPB/ DTPB, and combined TAM-TPB
	Social factors	MPCU
	Image	DOI
Facilitating conditions	Perceived behavioral control	TPB/DTPB and combined TAM-TPB
	Facilitating conditions	MPCU
	Compatibility	DOI

Created using source data from Venkatesh et al. (2003).

The article "Application and extension of the UTAUT2 model for determining behavioral intention factors in use of the artificial intelligence virtual assistants" was published in 2022. Journal: Front Psychol.

With UTAUT's underlying theoretical context, Venkatesh et al. (2012) provided a seminal framework to focus on the consumer viewpoint for an extended version UTAUT2, which aggregated three factors for considerations: *Hedonic Motivation, Price/value*, and *Habit*. This allows for a predictive capability built-into the model that substantially increases its potential for estimating user adoption up to 74% (Venkatesh et al., 2016). The applicable dimension of the theoretical approach had been well-established as a general framework within the technology industry. The large number of studies produced are evidence of a model that is fruitful for analysis in the new technologies' adoption areas and within innovative approaches, and as part of varying cultural and social contexts, gives us an enhanced framework for adoption (Šumak and Šorgo, 2016). Some fields of practical application and user, behavioral, and standard approach are often used for virtual classroom and learning (Dizon, 2021); banking and finances (Khan and Rabbani, 2021), and ecommerce (Biduski et al., 2020).

### Scientific research regarding virtual assistants

Many studies have approached user intention, as well as the factors for adoption in VA. Lu et al. (2021) focused on the context of Tourism and Hospitality from a defined consumer approach for long term integration of AI and robotics into common transactions around services for hotels, restaurants, airlines, and retail shop networks. From the analysis of lever factors, the variables that are rated as directly correlated to adoption, are: *PE, Intrinsic Motivation, (ergonomics), Social Influence, Facilitating Conditions*, and *Emotions*. Related to Tourism and Hospitality, the travel segment inspired another study focusing on devices for Intelligent Travel Assistants as these relate to eight variables impacting adoption, which are: *ease of use, trust, enjoyment, design, usefulness, quality, safety*, and *empathy*. External factors are showing an overall influence, such as, *usage, trust, hedonic motivation*, and *design*, to be followed by *utility, quality*, and *empathy*. In the institutional context and within organizations, the approach to study technology and VA adoption is taken from a task-oriented, work-environment approach. Some of the factors determining how satisfactory work conditions for a person can be, stem from technology use, as it is impacting productivity and level of tasks completion (Marikyan et al., 2022). In this context, the results point at *Performance Expectancy, Perceived Enjoyment, Social Presence*, and *Trust*, as positive factors directly impacting productivity and commitment from workers. Research conducted by McLean and Osei-Frimpong (2019), combined the theoretical underpinnings of Uses and Gratifications Theory (U&GT) with technological theories to obtain a clearer understanding of user motivations in their intent and use of voice assistants around the home. This research establishes a moderating role for the *Perceived Privacy Risks* that can diminish and negatively influence the use of voice assistants in the home. The results indicate the importance of the benefits that these devices grant us, since it will motivate the use of a voice assistant at home. Yang and Lee (2019) explain the intent and use of VA devices through *Perceived Utility, Perceived Enjoyment*, and product design-related, ergonomic, features. The results show that the *Perceived Usefulness* and *Enjoyment* have a significant impact on users' intention. From a hedonic value perspective, the content quality, which is also a functional attribute of VA devices, as well as visual appeal, positively affect *Perceived Enjoyment*.

The article "Application and extension of the UTAUT2 model for determining behavioral intention factors in use of the artificial intelligence virtual assistants" was published in 2022. Journal: Front Psychol.

UTAUT 2 has been used in diverse fields from widespread contexts. Vimalkumar et al. (2021) analyzed the factors that motivate people to use voice assistants for the home, adding other variables to the original set: *Perceived Privacy concerns, Perceived Privacy Risk*, and *Perceived Trust*. In the Kessler and Martin (2017) research, they identify the perceptions and determinants of potential future users linking to VA technology by adding the variables *Data Security, Compatibility*, and *Relationship* with the device to the framework model. Kalinić et al. (2019) analyzes the disposition of customers to use smart speakers for online purchases, adding the *Perceived Risk* variable to the model (Malarvizhi et al., 2022). Almahri et al. (2020) examines the factors that can deter or facilitate the acceptance and use of chatbots by university/college students in post-secondary education. Gansser and Reich (2021) analyzes factors influencing the use of VAs in a daily life environment in three segments of mobility, home, and health, adding the variables *wellbeing* and *health, convenience, comfort, sustainability, safety* and *security*, and *Personal Innovation*. Schmitz et al. (2022) investigated patients' intention in order to take advantage of virtual medical appointments by adding *Perceived Security*, and *Perceived Product Advantage* to the user intention model of variable analysis.

The article "Application and extension of the UTAUT2 model for determining behavioral intention factors in use of the artificial intelligence virtual assistants" was published in 2022. Journal: Front Psychol.

## Selected variables for the study

### Performance expectancy

The PE has been defined as “the degree to which the use of a technology will provide benefits to consumers in carrying out certain activities” (Venkatesh et al., 2003, p. 447). Therefore, it denotes the degree to which an individual perceives that virtual assistant can facilitate greater performance and productivity. Being a relatively recent technology, one foreseeable barrier was set at the possibility of visualizing potential for added tasks within the VA platform. The effect of this variable, on the attitude toward the use of technology, has been well-documented in previous literature on virtual assistants (Cyr et al., 2007; Hassanein and Head, 2007; Moriuchi, 2019; Ye et al., 2020). From this perspective, PE reflects the extrinsic degree of motivation or the expected result of the use. Previous research has seen this variable for its influence on the adoption of VA (McLean and Osei-Frimpong, 2019; Wagner et al., 2019; Koon et al., 2020; Vimalkumar et al., 2021). Therefore, based on this, the following hypothesis is proposed:

H1: PE positively and directly influences user's intention to use VA.

### Effort expectancy

EE is “the degree of ease associated with using the system” (Venkatesh et al., 2003, p. 450). In context it refers to the perceived ease in VAs usage. This factor is considered a fundamental predictor of technology adoption in research settings (Wirtz et al., 2019). When interacting with AI-based VAs, EE will appear to be implicit in most cases, being a barrier if they are not provided to the level expected by consumers (Wirtz et al., 2018, 2019) or require a high effort, since VAs have to allow consumers to execute tasks with minimal effort (McLean and Osei-Frimpong, 2019). The objective is therefore to have users achieve a positive perception regarding the “degree of ease” (Venkatesh et al., 2012), Previously it has been shown that confidence in one's own abilities to deal with technical systems has a significant influence, directly impacting the intention to use them (Fridin and Belokopytov, 2014). Previous research has studied this variable to understand its influence on VAs' adoption (Chopra, 2019; Zaharia and Würfel, 2020; Mishra et al., 2021; Moriuchi et al., 2021). Therefore, based on this it is hypothesized that:

H2: EE positively and directly influences user's intention to use VA.

### Social influence

SI is “the extent to which consumers perceive their significant others (like family and friends) believe they should use a particular technology” (Venkatesh et al., 2003, p. 451). In the context of the study, it is the degree to which an individual believes that important people support their use of VAs for their daily tasks. The SI based variable models an individual's beliefs and behavior through the interactional mechanisms of compliance, internalization, and identification (Moriuchi, 2021). Previous studies have provided empirical support that evidences the impact of SI on the use of technology in different contexts (Moriuchi, 2021). They have also studied this variable to examine its influence on the adoption of VAs (Chopra, 2019; Zaharia and Würfel, 2020; Mishra et al., 2021; Moriuchi et al., 2021). In this context our proposed hypothesis is the following:

H3: SI positively and directly influences user's intention to use VA.

The article "Application and extension of the UTAUT2 model for determining behavioral intention factors in use of the artificial intelligence virtual assistants" was published in 2022. Journal: Front Psychol.

### Facilitating conditions

*Facilitating conditions* are “consumers' perceptions of the resources and support available to perform a behavior” (Venkatesh et al., 2003, p, 453). Underlying this perception, there is the idea of acceptance; an information system depends on a preliminary assessment of one's own ability to master the new technology (Wong et al., 2020). Users need to perceive the presence of a solid support infrastructure that facilitates the learning and usage of the technology, so the usefulness of a technological device will be executed under the premise that facilitating conditions are actively working on a given environment (Canziani and MacSween, 2021). This scenario is particularly true in the context of AI-based technology, whether for individual or organizational use; it is necessary to have infrastructure that facilitates use (Grover et al., 2020). Vimalkumar et al. (2021) confirmed the positive influence of *facilitating conditions* on consumer adoption of digital voice assistants. In addition, previous research analyzed FC from the standpoint of influence on adoption, specifically, VAs (Gunasinghe et al., 2020; O'Connell et al., 2021; Al Shamsi et al., 2022) where the findings point at confirming the presence of this variable, thus:

H4: FC positively and directly influences user's intention to use VA.

### Hedonic motivation

HM is “the fun element, joy, or pleasure derived from the use of a particular technology without any specific additional benefit” (Venkatesh et al., 2012, pp. 157–178). Some authors state that HM is a key factor in consumer behavior (Holbrook and Hirschman, 1982), and that aspect linked to the fun and pleasure derived from usage, can be seen as crucial when evaluating, in advance, acceptance and technology use (Childers et al., 2001; Brown and Venkatesh, 2005). The greater the fun and pleasure elements anticipated from the use of a technology, the more likely consumers are to accept it. Understanding *hedonic motivation* for technology use relies on the assumption that arousal inherently makes people excited and more willing to accept and use something new—a natural tendency to initiate actions, that makes individuals, joyful, positive, and helpful. Previous research has analyzed this variable in experiences and VA adoption (Gunasinghe et al., 2020; O'Connell et al., 2021; Al Shamsi et al., 2022), and it has established that:

H5: HM positively and directly influences user's intention to use VA.

The article "Application and extension of the UTAUT2 model for determining behavioral intention factors in use of the artificial intelligence virtual assistants" was published in 2022. Journal: Front Psychol.

### Price/value

PV has been defined as “consumers' cognitive trade-off between the perceived benefits of apps and the cost of using them” (Venkatesh et al., 2012, pp. 157–178). Therefore, PV is a measure of the net benefit obtained by using a technology. In fact, people are always out to maximize net profit. This implies that, if the adoption and use of technology generate positive gains, individuals will accept the cost of it. Previous studies have confirmed the effect that price/value has on technology adoption, a process that is enhancing in itself, and as such, provides a positive feeling and impact on users (Moorthy et al., 2019; Palau-Saumell et al., 2019). In addition, the studies confirm that price/value and behavioral intention are closely related in positively improving intentional behavior and adoption due to the novel perception that it increases satisfaction (Moorthy et al., 2019; Palau-Saumell et al., 2019). Based on this variable and similar experiences in technology adoption for VAs (Ashfaq et al., 2021; Ling et al., 2021; Twum et al., 2021), the general conception is toward seeing:

H6: PV positively and directly influences user's intention to use VA.

### Habit

The HB is “the extent to which individuals tend to perform behaviors automatically due to learning” (Venkatesh et al., 2012, p. 157–178). As a consequence of repeated performance, when people internalize habits, they may not think about, realize, or evaluate the reasons for their actions (Mittal, 1988; Ouellette and Wood, 1998). In the context of VAs based on machine learning, habit allows the formation of a symbiotic relationship between the user and the technology (Jacucci et al., 2014). Hence, habit is not only an explanation of daily routines (Yen and Wu, 2016), but also an important factor that will determine the degree of user engagement with this type of technology (Perez-Vega et al., 2021). Previous research has analyzed this variable to study its influence on the adoption of VA (Kessler and Martin, 2017; Gunasinghe et al., 2020; Twum et al., 2021). Therefore, based on this the following hypothesis is suggested:

H7: HB positively and directly influences user's intention to use VA.

The article "Application and extension of the UTAUT2 model for determining behavioral intention factors in use of the artificial intelligence virtual assistants" was published in 2022. Journal: Front Psychol.

### Perceived privacy risk

*Perceived Privacy Risk* indicates the degree of perceived certainty of consumers that their personal information is shared with an information system (Lee et al., 2021). Therefore, privacy implies not being subjected to unwanted intrusions (Merriam-Webster and Springfield, 2005), such as wiretapping, the exploitation of security vulnerabilities and user identity theft (Chung et al., 2017). VAs cause a growing concern about privacy and security that are impediments to their use and adoption (Saura et al., 2021; Vimalkumar et al., 2021). Since VAs need to collect sensitive and private data for proper operation, security issues are raised for, and this fact entails a barrier to, their full adoption (Pitardi and Marriott, 2021). Previous research has examined how privacy concerns influence consumer responses in a variety of settings (Pizzi and Scarpi, 2020). These studies provide evidence that privacy concerns can act as an inhibitor (Nepomuceno et al., 2014). Thus, based on previous research and following its impact on adoption around VAs, our hypothesis is the following:

H8: Perceived Privacy Risk negatively and directly influences user's intention to use VA.

### Trust

*Trust* is generally conceived as a multidimensional concept that reflects perceptions of competence, integrity, and benevolence of another entity (Mayer et al., 1995). *TR* has been recognized as a key influencer of human-machine interactions (McLean et al., 2020). It builds on your perception of trustworthiness, which is enhanced by having faith in your interactions (Hengstler et al., 2016). *TR* is one of the most important elements to overcoming uncertainty (Yang and Lee, 2019). When technology is emerging, users often feel uncertain due to a lack of information. However, when users have a pre-existing feeling of trust toward a specific technology, a brand, or rely on referrals, this uncertainty can be eliminated. *TR* has been extensively researched in the VA field (Kuberkar and Singhal, 2020; Pitardi and Marriott, 2021; Vimalkumar et al., 2021). Previous research on *TR* highlights the role of technical features of websites and technology, such as ease of navigation, visuals, and ease of search, as signals that convey trustworthiness (Corritore et al., 2003). Prior research has analyzed this variable to study its influence on the adoption of VA (Kasilingam, 2020). Therefore, based on this our hypothesis is the following:

H9: TR positively and directly influences user's intention to use VA.

### Personal innovativeness

This is the area of adaptation to technology with a higher interest from a behavioral intention standpoint—for individuals to display a high degree of adoption of new products within a set user-base or a specific community (Juaneda-Ayensa et al., 2016; Getnet et al., 2019). In the area of VA adoption, innovation is measured in terms of function, hedonic motivation, and cognitive motivation. The effect of such variables toward adoption in VA has been studied in previous research to present a thesis for positive rate with an effect on adoption. Previous research recognizes this variable for its influence on the adoption of VA (Kasilingam, 2020; Hasan et al., 2021; Winkler, 2021). In this context, the last hypothesis is:

H10: PI positively and directly influences user's intention to use VA.

The article "Application and extension of the UTAUT2 model for determining behavioral intention factors in use of the artificial intelligence virtual assistants" was published in 2022. Journal: Front Psychol.

Figure 1 presents the developed research model.

**Figure 1:** The research model.

## Methodology

### Plan-design for data

The developed questionnaire for an effective market survey consists of two parts: (1) the instrument proposed by Venkatesh et al. (2012) to the context of Virtual Assistants with 24 questions that measure the 7 constructs of the UTAUT2; and (2) the questions of scholarly articles were adapted with 12 questions that measure the three factors added to the model. In addition, sociodemographic information is collected for contrasting data (Tables 2, 3). The 5-point Likert scale method is used, ranging from 1 (totally disagree) to 5 (totally agree). This scale avoids cognitive biases and the confusion of the respondents. In addition, it provides quality data, and it is recommended by researchers (Revilla et al., 2014). The structural equation model (SEM) was used for the analysis of the results, since it allows testing all the relationships between the observed and latent variables simultaneously, by combining multiple regression with factor analysis and provides general adjustment statistics (Iacobucci, 2010). In addition, it is capable of considering the measurement error with the observed variables (Hair et al., 2006).

**Table 2:** Variables for analysis.

**ID**	**Constructs**	**Items**	**Source**
1	Performance expectancy	4	Venkatesh et al., 2003
2	Effort expectancy	4	
3	Social influence	3	
4	Facilitating conditions	4	
5	Hedonic motivation	4	
6	Price/value	3	Venkatesh et al., 2012
7	Habit	3	
8	Perceived privacy risk	4	Featherman and Pavlou, 2003
9	Trust	3	Lu et al., 2011
10	Personal innovativeness	4	Agarwal and Prasad, 1998; Thakur and Srivastava, 2014
11	Behavioral intention	3	Venkatesh et al., 2003

**Table 3:** Survey questions.

**Constructs**	**Items**	**Question**
Performance expectancy	PE1	Voice assisted devices appear useful for everyday common tasks…
	PE2	Voice assisted devices supplemented options for completing tasks that are essential to me…
	PE3	Voice assisted devices aided in completing tasks faster…
	PE4	Voice assisted devices increased productivity for…
Effort expectancy	EE1	In order to learn new information, voice assisted devices provided an easier means to…
	EE2	My interaction with voice assisted devices features a clear sound and easy to understand speech…
	EE3	I find that voice assisted devices are easy to use…
	EE4	It is easy for me to feel competent around voice assisted devices…
Social influence	SI1	People that are close to me consider that using voice assisted devices is…
	SI2	People that affect my everyday life and have an effect on my personal choices, consider that I should use voice assisted devices…
	SI3	People with opinions that are valuable to me have a preference for voice assisted devices…
Facilitating conditions	FC1	I have access to the necessary resources in order to be able to use voice assisted devices…
	FC2	I have the basic level of skill in order to be able to use voice assisted devices…
	FC3	Voice assisted devices are compatible with other devices that I already use…
	FC4	I am able to get online support for any difficulty arising during times when I use voice assisted devices…
Hedonic motivation	HM1	Using voice assisted devices is fun…
	HM2	Using voice assisted devices is enjoyable…
	HM3	Using voice assisted devices is entertaining…
Price/value	PV1	Voice assisted devices are reasonably priced…
	PV2	I am willing to pay for using platforms associates with the use of voice assisted devices…
	PV3	The cost for services added to voice assisted devices is manageable and it fits with added benefits…
Habit	HB1	Using voice assisted devices is fun…
	HB2	Using voice assisted devices is enjoyable…
	HB3	Using voice assisted devices is entertaining…
Trust	TR1	Voice assisted devices are trustworthy…
	TR2	I trust voice assisted devices for their ability to perform its functions…
	TR3	Voice assisted devices are capable of performing assigned tasks…
	TR4	Voice assisted devices in still trust in me…
Perceived privacy risk	PSE1	I have concerns about personal data protection and privacy whenever I use voice assisted devices…
	PSE2	I have concerns for security and data protection whenever I use Voice assisted devices…
	PSE3	I have concerns around privacy associated with the systems' use around voice assisted devices…
	PSE4	I have concerns around security issues associated with the systems' use around voice assisted devices…
Personal innovativeness	PI1	I like experimenting with voice assisted devices…
	PI2	I am generally an early user among colleagues and active user of voice assisted devices…
	PI3	Generally, I am hesitant to try the new voice assisted devices…
	PI4	I would seek new ways and experiment with voice assisted devices…
Behavioral intention	BI1	I intent to use voice assisted devices in the future…
	BI2	I will continue to use voice assisted devices regularly in my everyday life…
	BI3	My plan is to continue on using voice assisted devices often…

The article "Application and extension of the UTAUT2 model for determining behavioral intention factors in use of the artificial intelligence virtual assistants" was published in 2022. Journal: Front Psychol.

### Data collection

After completing the pilot test to clarify phrasing and eliminate items that were not identifiable in the questionnaire, the empirical data was obtained from the questionnaire and executed through a Google form that was *distributed online and in person, via* door-to-door survey to individuals in post-secondary campuses and in other urban districts, by using a QR code; it was implemented during the first quarter of 2022. Non-probabilistic convenience sampling was used. Three hundred and six responses were obtained. A first descriptive analysis using IBM SPPS Statistics 27 examined the data for missing pieces of information, uncommitted responses, outliers, and for data leveling. There were no missing data in the set. Thus, in Table 4 a descriptive sociodemographic data of the sample is presented.

**Table 4:** Survey feature profile.

**Variable**	**Description**	**Frequency**	**Percentage %**
Gender	Female	189	61.8
	Male	117	38.2
	Prior to 1965	19	6.2
Year of birth	1965–1979	35	11.4
	1980–1999	90	29.4
	After 2000	162	52.9
Level of education	Elementary school	0	0.30
	Higher secondary school	5	1.6
	Bachelor	147	48
	High education	154	50.3
Use virtual assistants	Yes	230	75.2
	No	76	24.8
Frequency use virtual assistants (Last month)	0	63	20.6
	1–10	172	56.2
	11–20	36	11.7
	over 21x	35	11.5
Use of virtual assistants as only option	Yes	62	20.3
	No	244	79.7

### Data analysis

#### Modeling analysis: Framework

Prior to the estimation analysis of the models the Mardia coefficient was calculated, which showed the multivariate non-normality of the data obtained, since it should not exceed the value 70. The results show a Kurtosis = 221.443 and a critical region = 29.693; however, considering that the skewness coefficients were <3 and the kurtosis coefficients <10, the maximum likelihood procedure was continued. A confirmatory factor analysis CFA test was performed using SPSS 27 and AMOS 27 tools to verify the measurement model by examining convergent validity, discriminant validity, and internal consistency of the constructs. To estimate convergent validity, the following were measured: the reliability of the measurement item (factor load), the reliability of each construct CR, and the average variance extracted AVE (Anderson and Gerbing, 1988). The values of the standardized factor loadings ranged between 0.588 and 0.933, which is higher than the required value of 0.50 (Gefen et al., 2000). Meanwhile, the composite reliability values demonstrated internal consistency of the latent constructs with values above the threshold of 0.70 (Heinzl et al., 2011). Finally, the values of the average variance extracted AVE, which are a measure of the variation explained by the latent variable to the random measurement error, ranged between 0.557 for *performance expectation* and 0.81 for *social influence*, above the lower stipulated limit of 0.50 (Fornell and Larcker, 1981). Therefore, all the predictors in this study, as can be seen in Table 5, are highly reliable, and the convergent validity results suggest that the latent constructs are good within the observed variables, since they are correlated with each other within the bottom-line model.

The article "Application and extension of the UTAUT2 model for determining behavioral intention factors in use of the artificial intelligence virtual assistants" was published in 2022. Journal: Front Psychol.

**Table 5:** Results for the measurement model.

**Constructs**	**Items**	**Standard loadings**	**CR**	**AVE**
Performance expectancy	PE1	0.864	0.833	0.557
	PE2	0.652		
	PE3	0.715		
	PE4	0.74		
Effort expectancy	EE1	0.868	0.914	0.727
	EE2	0.77		
	EE3	0.887		
	EE4	0.88		
Social influence	SI1	0.875	0.927	0.81
	SI2	0.933		
	SI3	0.89		
Facilitating conditions	FC1	0.866	0.888	0.669
	FC2	0.901		
	FC3	0.853		
	FC4	0.62		
Hedonic motivation	HM1	0.907	0.91	0.77
	HM2	0.9		
	HM3	0.824		
Price/value	PV1	0.853	0.922	0.798
	PV2	0.94		
	PV3	0.885		
Habit	HB1	0.872	0.842	0.646
	HB2	0.614		
	HB3	0.894		
Trust	TR1	0.77	0.863	0.612
	TR2	0.79		
	TR3	0.774		
	TR4	0.796		
Perceived privacy risk	PSE1	0.889	0.863	0.765
	PSE2	0.933		
	PSE3	0.685		
	PSE4	0.588		
Personal innovativeness	PI1	0.737	0.855	0.597
	PI2	0.697		
	PI3	0.805		
	PI4	0.842		
Behavioral intention	BI1	0.84	0.894	0.738
	BI2	0.82		
	BI3	0.91		

For the evaluation of discriminant validity, Heterotrait-Monotrait (Henseler et al., 2015) is used as an estimator of the correlation between two latent variables. According to this indicator, the coefficients must be below 0.90, in all cases they offered levels below 0.90, as can be seen in Table 6, which confirms the discriminant validity of all the latent used variables. For this, the construct measured items were required and they did not interlink with other concepts.

**Table 6:** Ratio heterotrait-monotrait.

	**PE**	**EE**	**SI**	**FC**	**HM**	**PV**	**HB**	**PI**	**PSE**	**TR**	**BI**
PE											
EE	0.544										
SI	0.67	0.29									
FC	0.434	0.873	0.229								
HM	0.562	0.725	0.336	0.732							
PV	0.399	0.319	0.341	0.323	0.44						
HB	0.785	0.425	0.629	0.339	0.441	0.59					
PI	0.61	0.256	0.549	0.182	0.4	0.39	0.675				
SS	0.2	0.097	0.164	0.06	0.068	0.21	0.142	0.215			
T	0.611	0.634	0.429	0.611	0.593	0.47	0.556	0.593	0		
B	0.796	0.534	0.582	0.494	0.59	0.48	0.83	0.788	0.104	0.78	

The general fit of the measurement model (Figure 2) to assess quality was performed through the evaluation of four goodness-of-fit indicators: the divided chi-square fit index PCMIN/DF, comparative goodness-of-fit index CFI, root of the residual root mean square of approximation RMSEA, and p of Close Fit (PCLOSE). The measurement model is considered sufficiently adjusted when these measurements are <3, ≥0.95, ≥0.90, ≤0.06 (Hair et al., 2006). The results: (PCMIN/DF 2.154, CFI 0.896, RMSA 0.050). This confirms that the measurement model has a high goodness of fit to (level) the data.

The article "Application and extension of the UTAUT2 model for determining behavioral intention factors in use of the artificial intelligence virtual assistants" was published in 2022. Journal: Front Psychol.

**Figure 2:** Measurement model.

#### Structural model assessment

##### Data set sample validation

With the aim of validating the adequacy of samples collected, Hoelter's N critical index was applied with a significance level of 0.05, equivalent to 95% confidence (Hoelter, 1983; Bollen and Liang, 1988). The appropriate threshold for a good fit is 200, and values below 75 are considered unacceptable (75 ≤ value < 200; acceptable ≥ 200) (Wan, 2002; Garson, 2014). The size of the sample with 230 questionnaires is acceptable, since the Holter analysis concluded that the minimum size necessary for the sample would have been 117 questionnaires for a 95% reliability.

##### Framework-model analysis

Four common measures of model fit were used to assess the overall goodness of fit of the model. The results of the proposed research model showed an adequate fit: (PCMIN/DF 2.154, CFI 0.896, RMSA 0.050). The next step in evaluating the structural model (Figure 3) is to measure the explanatory power of the dependent variable measured as R-squared *R*^2^. This is used as a measure of the explanatory power of the model ensemble and describes how much of the dependent variable is explained by the independent variables in the model. *R*^2^ values range from 0 to 1. Values closer to 1 are indicative of more significant explanatory power, and values >0.9 are indicative of model overfitting that could cause inaccurate results. Behavioral user intention was found to have an *R*^2^ of 0.898, indicating that 89.8% of the variable was explained by the independent variables in the model. That is, the model elucidated an 89.8% for measuring the behavioral intention in the realm of VAs.

**Figure 3:** Final structural-model.

One final step entails evaluating the chain relation in the cause linking constructs *via* the structural model (Hair et al., 2010). The relation between independent variables and dependable prove a median, average beta coefficient (β), the statistics T and the value of *p*. The SEM results in Table 7 display the guidelines H7, H9, H10, as significant, vs. *habit, trust* and *personal innovation* as being significantly correlated with user intention in VA's. Also, we consider *habit* (β = 0.408, *p* < 0.001) a good predictor, being followed by *trust* (β = 0.291, *p* < 0.001), and in last place, lowered score for *personal innovativeness* (β = 0.267, *p* < 0.001). The guidelines H1, H2, H3, H4, H5, H6, and H8, *performance expectancy* (β = 0,136, *p* > 0.1), *effort expectancy* (β = −0.141, *p* > 0.1), *social influence* (β = −0.008, *p* > 0.1), *facilitating conditions* (β = 0.170, *p* > 0.1), *hedonic motivation* (β = 0.049, *p* > 0.1), *price/value* (β = −0,76, *p* > 0.1) and *perceived privacy risk* (β = 0.002, *p* > 0.1) user intent does not represent a meaningful thrust in the context of a Spanish VAs user-base.

The article "Application and extension of the UTAUT2 model for determining behavioral intention factors in use of the artificial intelligence virtual assistants" was published in 2022. Journal: Front Psychol.

**Table 7:** Results.

**Guidelines**	**β**	***t-*** **value**	***p*** **-value**	**Decision**
H1: Performance expectancy **→** Behavioral intention	0.136	1.368	0.171	Unsupported
H2: Effort expectancy **→** Behavioral intention	−0.141	−1.230	0.219	Unsupported
H3: Social influence **→** Behavioral intention	−0.008	−0.150	0.881	Unsupported
H4: Facilitating conditions **→** Behavioral intention	0.170	1.522	0.128	Unsupported
H5: Price/Value **→** Behavioral intention	−0.76	−1.461	0.144	Unsupported
H6: Habit **→** Behavioral intention	0.408	4.177	^***^	Supported
H7: Hedonic motivation **→** Behavioral intention	0.049	0.720	0.471	Unsupported
H8: Perceived privacy risk **→** Behavioral intention	0.002	0.573	0.958	Unsupported
H9: Trust **→** Behavioral intention	0.291	0.052	^***^	Supported
H10: Personal innovativeness **→** Behavioral intention	0.267	3.751	^***^	Supported

Measurement correlation-values:

*** *p* < 0.001.

## Results and discussion

What are the factors impacting users' intention and VAs usage? The model framework UTAUT2 establishes an empirical base for several constructs and suggests that behavioral user intention responds to *habit, trust*, and *personal innovation*. The model assigns 89.8% of predictability to user intention. From the model analysis it is established that PE (H1), doesn't impact intention of usage. Despite a number of studies pointing at PE and benefit perceived in VAs toward higher adoption rate (Fan et al., 2022) for providing a pleasurable experience (Tsay and Patterson, 2018), that in turn will add to intention of use and to adoption rates (Almaiah et al., 2019), for the present case scenario didn't show a significant impact toward an increase in user perception or an improved expectation for performance. This bottom line is backed up by the referenced studies (Khalid et al., 2021; Pitchay et al., 2021). From a user skill consideration of VAs usage and adoption, most participants in the 52% spectrum were millennials and digital natives, so, functioning and display of simple commands, searches, and chat natural to the interface did not require any upgrades for the users' technical knowledge (Melián-González et al., 2021). Thus, this factor is irrelevant to EE by minimizing setting up and action-tasks specific to VA usage. Ease of use as a non-relevant factor has been established in several studies (Wirtz et al., 2018, 2019; Zarouali et al., 2018; Balakrishnan and Dwivedi, 2021; Lv et al., 2021; Aw et al., 2022; Moussawi et al., 2022).

The article "Application and extension of the UTAUT2 model for determining behavioral intention factors in use of the artificial intelligence virtual assistants" was published in 2022. Journal: Front Psychol.

Aligned with ease-of-use factors arising from SI, we can take into account that colleagues and close individuals provide a referential standard from a common core belief and a similar mindset toward technology adoption. For the geographical scope of the study, Spain's population without wider access to technology will not have an impact in usage. Presence on apps and smart platforms of VAs, such as Alexa, Siri, and Cortana, extends to 16.9% of the total population in Spain (Survey in TIC Hogares, 2020). For use of VAs, specific targets show a 9.4% frequent use, several times a day, while a 6.1% use them once a day (Statista, 2022). This low rate of penetration clearly links to a lower degree of influence within a network, as shown by previous research (Hu et al., 2019).

FC (H4) did not affect usage or behavioral intent, considering that individuals have the necessary skill and ability in order to use VAs without additional technical support. Then, *facilitating conditions* are not essential contributing causes used to deter or favor user intention as shown in scholarly research (Alalwan et al., 2017), bearing in mind that ease of use specific to assistant devices does not imply a need for structural support to install the platform or to use the application.

VA adoption is not impacted by a *hedonic motivation*, seeing that the most common tasks, searches, and easy questions, are accessible *via* these assistants to most Spanish users according to an AIMC Study (2021). The distribution of tasks in this category presents the areas of interactions that are most common—searches/questions, weather/traffic report, music streaming and internet radio, alerts, calendar reminders, to-do-lists, call display, newscasts, messaging, central control for home appliances, shopping/online orders/meal delivery providers—a landscape of everyday applications that aligns with previous research (Laumer et al., 2019; McLean and Osei-Frimpong, 2019; McLean et al., 2021).

*Price/value* (H6) is not a significant factor due to an added advantage originating in zero cost for installation and from the perception of affordability to access technology assisting devices, such as, central speakers.

The article "Application and extension of the UTAUT2 model for determining behavioral intention factors in use of the artificial intelligence virtual assistants" was published in 2022. Journal: Front Psychol.

Contrary to *price/value* as it relates to ease of use, *habit* (H7) has a significant effect over intention of use in the VAs segment. As part of social psychology, habits include learned actions, mnemonic rules, and repetition of sequences from experiences in the same way specific actions create a consistent, recurrent, and pattern in results (Verplanken and Faes, 1999). Therefore, an automated action will be completed with the expectation of a known incentive. The more an action yields a specific result, associated to a benefit, the more this link forms between action and reward, thus carrying a behavior over time and without added effort (Lally and Gardner, 2013). From this perspective, the younger generation, having breath from a digital environment where they depend on mobile devices and apps for most of their everyday tasks, are inherently competent and naturally fall in the path of automation when using VAs. By integrating the string of tasks listed as simple access to assistants, these devices become integrated, as well as contributing to the development of digital skills of VA (Kessler and Martin, 2017; Gunasinghe et al., 2020). This positive influence stands against other scholars' analysis with negative findings around the impact of HB in usage (He et al., 2022).

Our framework and data analysis supported that *privacy risks* (H9) do not impact user intention. In the VAs' area, the risks associated with security and privacy are aligned with third-party access to unauthorized, restricted information bands, and consequent data-breaches around personal information in the system (Han and Yang, 2018). One added benefit of a VA is listening to and storing requests; however, the security layer provides a perception risk in a manner that is not entangled with “trustworthiness” or “authorized access.” Additionally, the compilation of personal information entrusted into the privacy of the system would not add a layer of risk when the service provider stores information according to set standards for security. This could be detrimental to the overall factors impacting adoption, but it is not a barrier in the use of an assistant device; the added risk is powerful among perceived situation or potential risks, but it isn't perceived or felt as such by users during their interactions who relied on the ease of use and its practicality.

This gap existing between the will to shield or share data is measured by trust. *Trust* (H9) changes toward the service and the provider of a platform. The service provided is established between individuals at the time of performing a task when the expectation is placed on the system responding to the present interaction and communicating the results fast and efficiently, in a reliable manner. On one hand, trust in the service provider links to credibility and established reputation. Some technology platforms providing service access to servers are Amazon, Google, and Apple—companies with a long-known trajectory and degree of trust that will eliminate initial user resistance toward enrolling in one of these service provider platforms. On the other hand, lack of trust will yield a lower adoption rate in the specific segment of VAs, due to underlying risks to privacy and trust, conducive to technology distrust (Cho et al., 2020; Zierau et al., 2020); accordingly, design of interface should be sensitive to this layer of risk and trust (Cho et al., 2020; Chen et al., 2021). Consistent with this line of thought, trust is a known factor in studies for user acceptance of VAs (Kuberkar and Singhal, 2020; Pitardi and Marriott, 2021; Vimalkumar et al., 2021).

The article "Application and extension of the UTAUT2 model for determining behavioral intention factors in use of the artificial intelligence virtual assistants" was published in 2022. Journal: Front Psychol.

Personal innovation influences behavioral intention, and for many researchers working in this variable, it is most promising in arising technologies, since leading into a role within a known process will cause an evolution into more immediate acceptance than other individuals that are lacking involvement with new technologies. This assertion reinforces the belief that innovative people are capable of remaining optimistic and positive when confronted with new technology developments (Dabholkar and Bagozzi, 2002). This is consistent with preliminary standards confirming PI as having a high degree of influence in a user's intention (Kasilingam, 2020).

## Conclusions and implications

After the pandemic COVID-19 virus, many geographical areas showed an increase in VAs usage. There are few studies for reference after the global health crisis, and this model for analysis and study aims at filling this gap in the research of factors influencing introduction of new devices for virtual assistants. From a quantitative standpoint, there is a new methodology showing user intention around VAs' use and adoption in Spain. An underlying factor contributing to this context, arose from previous studies; based on AI introduction and a wide, all encompassing approach, to technology adoption (Wirtz et al., 2018, 2019); these changes have widened the scope in the theory and framework for analysis, to apply new filters for assessment of *trust, privacy risk*, and *personal innovation* in VAs. The information provided toward personal user experience can provide guidance for any development in the technological areas of health, business, home smart-systems (energy, security), and personalized bots-assistant companion. Considering that expanded use of the VA in these varied facets from industry to household, involve a massive potential for growth, this theoretical contribution and data analysis brings new light into personal innovation as a seminal variable for an integrated framework, with a focus on the interdependency of technology use and its context, limited to a national framework, the Spanish territory.

The article "Application and extension of the UTAUT2 model for determining behavioral intention factors in use of the artificial intelligence virtual assistants" was published in 2022. Journal: Front Psychol.

The above considerations are relative to the degree of technology development, skill, and competence around technology use as well as individual perceptions on the new applications (Alalwan et al., 2018). For the time-period framework, narrowed down to the years of global pandemic and defined by a health regulated environment, the study contributes data foreshadowing the novel role of consumer devices within a Spanish demographic, targeting device usage in diverse areas of daily life, from entertainment and home assistance to deliveries (Guzman, 2019). A second aspect under consideration is the effect of technology innovations as part of a context sensitive to added security and perceived risks; whether these devices make life easy without an added cost to privacy is a variable that opens a holistic sense into understanding the use of VAs as this field is evolving along AI. Personal innovation gains an edge for an integrated framework with essential notions established from behavioral intention. This notion is proposed by Dinev and Hart (2006) and proves to be productive in creating a cohesive base for analysis in line with a set of variables. In the area of VAs, personal innovation creates a filter valuable to system designers and business developers working in Vas as a means for retrofitting from clients, and to account for adoption with, an in-depth outlook into systems for prospecting of features and improvement processes (Kabra et al., 2017; Khalilzadeh et al., 2017). This is a valuable lesson obtained from the survey: it is important to have a customer centric approach, a user focus, along with a reputation for trustworthiness and low risk in bringing new features and generating innovations for an overall positive adoption rate. The information arising from the results represents a practical contribution looking forward into systems design and for businesses working in VA platforms. The data contrasted with an aligned set of variables will not only bring main factors that are relevant to user design to the discussion, but also highlight the need to integrate new features for increased trust, low risk, and greater innovation around digital assistants.

The article "Application and extension of the UTAUT2 model for determining behavioral intention factors in use of the artificial intelligence virtual assistants" was published in 2022. Journal: Front Psychol.

## Limitations and future research

There are some limitations of the present study even after reaching our set of objectives. Mainly, the results should be taken with caution for the limited scope of demographic data and only applied to the Spanish population. The same guidelines for ten factors of users' intention, can be extended for a cross-sectional approach to other geographical areas. Also, a cross-sectional study can be developed—an analytical approach from variables representing a synchronic set of standards for the data compiled in a specific timeframe—involving subjects and survey respondents' opinion evolution over time. Thus, results of the present analysis show that, indeed, *trust* leads to adoption, whereas *privacy risk* does not. Even though these factors are not new for studying users' adoption of the technological devices and smart technology, the context of application of the two factors leads researchers to open new paths for studies of continued use of VAs.

Finally, it could be appropriate to integrate new factors to the scope of variables and set of constructs, such as ergonomics, for dismantling an embedded bias around physical characteristics and their relation to mind processes, as these link to non-humans (for a technological viewpoint) with the aim of adding a layer of humanization to the process. This tendency to provide an animal form is known as anthropomorphism, which in turn, results in additional trust and satisfaction from a user, and even security, offering a more nuanced base for filtering of a subjective process. Prospective areas of development may bring a new insight on the link from intention to usage. Also, it may consider including other moderating variables for a study, such as gender, age, experience, and needs/desirable outcomes from use.

## Data availability statement

The original contributions presented in the study are included in the article/supplementary material, further inquiries can be directed to the corresponding author.

## Ethics statement

Ethical review and approval was not required for the study on human participants in accordance with the local legislation and institutional requirements. Written informed consent from the patients/participants or patients/participants legal guardian/next of kin was not required to participate in this study in accordance with the national legislation and the institutional requirements.

## Author contributions

MG: hypothesis proposal, data analysis, and manuscript preparation. JS: data collection. AA: manuscript revision. All authors contributed to the article and approved the submitted version.

## Conflict of interest

The authors declare that the research was conducted in the absence of any commercial or financial relationships that could be construed as a potential conflict of interest.

The article "Application and extension of the UTAUT2 model for determining behavioral intention factors in use of the artificial intelligence virtual assistants" was published in 2022. Journal: Front Psychol.

## Publisher's note

All claims expressed in this article are solely those of the authors and do not necessarily represent those of their affiliated organizations, or those of the publisher, the editors and the reviewers. Any product that may be evaluated in this article, or claim that may be made by its manufacturer, is not guaranteed or endorsed by the publisher.
